This article has been retracted.

# Suppression of microRNA-205-5p in human mesenchymal stem cells improves their therapeutic potential in treating diabetic foot disease

**DOI:** 10.18632/oncotarget.17012

**Published:** 2017-04-10

**Authors:** Lingyan Zhu, Gongxian Wang, Shane Fischbach, Xiangwei Xiao

**Affiliations:** ^1^ Department of Endocrinology, The First Affiliated Hospital of Nanchang University, Nanchang 330006, China; ^2^ Department of Urology, The First Affiliated Hospital of Nanchang University, Nanchang 330006, China; ^3^ Division of Pediatric Surgery, Department of Surgery, Children's Hospital of Pittsburgh, University of Pittsburgh School of Medicine, Pittsburgh, PA15224, USA

**Keywords:** diabetic foot disease (DF), microRNA, mesenchymal stem cells (MSCs), vascular endothelial growth factor (VEGF)

## Abstract

Diabetes is a prevalent disease endangering human health, while diabetic foot disease (DF) is one of the most severe complications of diabetes. Mesenchymal stem cells (MSCs) have been used in DF treatment, taking advantage of the differentiation potential of MSCs into endothelial cells and their production and secretion of trophic factors like vascular endothelial growth factor (VEGF). Molecular modification of MSCs to improve their therapeutic effects has been recently applied in treating other diseases, but not yet in DF. Here, we found that micoRNA-205-5p (miR-205-5p) is expressed in human MSCs, and miR-205-5p inhibits protein translation of VEGF through its interaction with 3′-UTR of the VEGF mRNA. Expression of antisense of miR-205-5p (as-miR-205-5p) significantly increased both cellular and secreted VEGF by MSCs, which significantly improved the therapeutic effects of MSCs on DF-associated wound healing in diabetic NOD/SCID mice. Together, our data suggest that miR-205-5p suppression in MSCs may improve their therapeutic effects on DF, seemingly through augmentation of VEGF-mediated vascularization.

## INTRODUCTION

The diabetic foot (DF) is one of the serious complications of diabetes, a prevalent disease with increasing incidence worldwide [1]. DF substantially delays normal cutaneous wound healing, leading to the need for amputations, as well as to substantial morbidity and mortality [1]. The diabetic state alters angiogenic homeostasis, leukocyte infiltration, macrophage function, extracellular matrix deposition and fibroblast transformation, which may affect all phases (coagulation, inflammation, re-epithelialization and remodeling) of wound healing [2]. Despite the complexity of the wound healing process and due to a number of defects in DF pathology, current treatment for DF focuses on promotion of revascularization through various growth factors, including vascular endothelial growth factor (VEGF) [3].

VEGF has been shown to significantly enhance the wound healing process in diabetic mice [4–6]. There are 6 members in the VEGF family, named VEGF-A/B/C/D/E and placental growth factor. The most potent pro-angiogenic factor in VEGF family is VEGF-A, which is simplified as VEGF in the scope of the current study. We have previously shown that VEGF release and production are independently regulated in pancreatic beta cells and duct cells, which are critical for physiological control of beta cell mass [7, 8].

Bone-marrow-derived mesenchymal stem cells (MSCs) are characterized by the potential to adhere to plastic, specific surface antigen expression (CD73+ CD90+ CD105+ CD34- CD45- HLA-DR-) as well as multipotent differential potential into cells of mesodermal origin, like adipocytes, osteocytes and chondrocytes, when the cells are kept *in vitro* differentiation conditions [9]. Since MSCs are well accessible and easily expanded *ex vivo*, MSCs have been used for cellular therapy involved in tissue repair and organ remodeling associated with DF, taking advantage of the differentiation potential of MSCs into endothelial cells and their production and secretion of vascular trophic factors like VEGF [10]. However, although genetic modification of MSCs has been shown to further improve their therapeutic effects on different diseases [11–13], genetic editing of MSCs to improve their therapeutic effects on DF has not been reported.

MicroRNAs (miRNAs) are non-coding small RNAs that control protein translation through Watson-Crick pairing to the 3′-untranslated region (3′-UTR) of the mRNA of a specific gene, resulting in alterations in protein translation and mRNA degradation [14]. The role of miR-205-5p in carcinogenesis has been well documented, in which many targets of miR-205-5p have been defined in cancer cells [15–19]. Very recently, VEGF has been found to be a target of miR-205-5p in glioma and miR-205-5p appears to be a glioma-specific tumor suppressor [20]. However, a role of miR-205-5p in regulation of the therapeutic potential of MSCs in DF has not been reported.

Here, we showed that miR-205-5p is expressed in human MSCs, and inhibits VEGF protein translation through its association with VEGF mRNA. Expression of antisense of miR-205-5p (as-miR-205-5p) significantly increased levels of cellular and secreted VEGF by MSCs *in vitro* and *in vivo*. MSCs depleted of miR-205-5p had increased therapeutic effects on DF in diabetic NOD/SCID mice.

## RESULTS

### Lower levels of VEGF and CD31 are detected in the resected DF specimens

The therapeutic effects of MSCs on DF substantially rely on their pro-angiogenetic effects. Indeed, in the resected DF specimens from the patients who received amputations, we detected significantly lower VEGF levels by ELISA (Figure 1A), and significantly lower levels of CD31, a specific endothelial cell marker, by Western blotting, compared to non-DF controls (Figure 1B). These data confirmed the presence of impairment in vascularization and lack of pro-angiogenic factors in DF, suggesting that increasing angiogenic potential of MSCs may enhance their therapeutic effects on DF.

**Figure 1:** Lower levels of VEGF and CD31 are detected in the resected DF specimens Resected DP specimens (*n* = 21) from the patients who received amputations were compared to comparable tissue from non-DF specimens (*n* = 17). (**A**) VEGF levels by ELISA (**B**) CD31 levels by Western blotting. *p < 0.05.

### Evidence of post-transcriptional control for VEGF by miR-205-5p in human MSCs

Next, we compared the VEGF mRNA and protein levels in human MSCs, compared to human endothelial cells (HUVEC). To our surprise, human MSCs expressed higher VEGF mRNA (Figure 2A), but lower cellular VEGF protein (Figure 2B) and lower secreted VEGF protein (Figure 2C), compared to HUVEC. We have previously demonstrated that VEGF synthesis and release may be differentially regulated in a cell-type-dependent manner. Here, the comparable levels of cellular and secreted VEGF suggest that the incomparable VEGF mRNA and protein may not result from the cellular control of VEGF release, but likely result from the post-transcriptional control of VEGF protein. Since miRNAs are important regulators for protein translation through their direct interaction with mRNA, we looked for the presence of such a regulatory miRNA for VEGF in MSCs.

**Figure 2:** Evidence of presence of post-transcriptional control for VEGF by miR-205-5p in human MSCs (**A**–**C**) VEGF levels in human MSCs were compared to HUVEC. (A) VEGF mRNA by RT-qPCR (B) VEGF cellular protein by ELISA (C) VEGF secreted protein in conditioned media by ELISA. (**D**) Bioinformatics analyzing results for VEGF-binding miRNAs expressed in MSCs with high “context++ score”. (**E**) Relative expression levels for 6 VEGF-binding miRNAs expressed in MSCs with high “context++ score”. (**F**–**H**) VEGF mRNA by RT-qPCR (F), VEGF cellular protein by ELISA (G) and VEGF secreted protein in conditioned media by ELISA (H) in MSCs transfected with antisense (as) for 6 VEGF-binding miRNAs expressed in MSCs with high “context++ score”. *p < 0.05. NS: non-significant. *N* = 5.

We performed bioinformatics analyses for miRNAs that bind to the 3′-UTR of VEGF mRNA. Among all VEGF-targeting miRNAs, we found 6 miRNAs that had high “context++ score” [21] (Figure 2D), expressed by human MSCs (Figure 2E). We thus inhibited expression of each miRNA in MSCs by transfection of the antisense of the corresponding miRNA. We found that the VEGF mRNA levels in MSCs were unchanged by transfection of either miRNA (Figure 2F). Moreover, the cellular VEGF protein (Figure 2G) and secreted VEGF protein (Figure 2H) were significantly increased only in miR-205-5p antisense (as-miR-205-5p)-transfected MSCs. These data suggest that miR-205-5p may be a VEGF-regulatory miRNA in MSCs.

### MiR-205-5p targets 3′-UTR of VEGF mRNA to inhibit its translation in MSCs

Indeed, bioinformatics analyses showed that miR-205-5p bound to 3′-UTR of VEGF mRNA at 150th-157th base site (Figure 3A). To confirm that this binding is functional, we transfected MSCs cells with plasmids carrying either as-miR-205-5p, or null as a control. Both plasmids co-expressed a RFP reporter. The transfected MSCs were purified based on RFP expression by flow cytometry (Figure 3B) and appeared red fluorescent in culture (Figure 3C). We found that transfection with as-miR-205-5p reduced miR-205-5p levels in MSCs by about 80% (Figure 3D). Although transfection by as-miR-205-5p did not alter VEGF mRNA in MSCs (Figure 3E), it significantly increased cellular VEGF protein (Figure 3F) and secreted VEGF protein (Figure 3G). Finally, a wildtype 3′-UTR of VEGF mRNA (VEGF 3′-UTR wt) plasmid, or a 3′-UTR of VEGF mRNA plasmid with mutant at the miR-205-5p-binding site (VEGF 3′-UTR mut), was used to co-transfect MSCs together with as-miR-205-5p or null plasmids in a dual luciferase reporter assay. While as-miR-205-5p significantly increased luciferase activity of VEGF 3′-UTR wt, the presence of a mutation abolished this effect (Figure 3H). Together, these results suggest that miR-205-5p may specifically target 3′-UTR of VEGF mRNA to inhibit its translation in MSCs.

**Figure 3:** MiR-205-5p targets 3′-UTR of VEGF mRNA to inhibit its translation in MSCs (**A**) Bioinformatics prediction of binding site of miR-205-5p on 3′-UTR of VEGF mRNA (150th-157th base site). (**B**–**C**) MSCs were transfected with plasmids carrying either as-miR-205-5p, or null as a control. Both plasmids co-expressed a RFP reporter. The transfected MSCs were purified based on RFP expression by flow cytometry (B) and appeared red fluorescent in culture (C). (**D**) RT-qPCR for miR-205-5p in null- or as-miR-205-5p-transfected MSCs. (**E**–**G**) VEGF mRNA by RT-qPCR (E), VEGF cellular protein by ELISA (F) and VEGF secreted protein in conditioned media by ELISA (G) in null- or as-miR-205-5p-transfected MSCs. (**H**) A wildtype 3′-UTR of VEGF mRNA (VEGF 3′-UTR wt) plasmid, or a 3′-UTR of VEGF mRNA plasmid with mutant at the miR-205-5p-binding site (VEGF 3′-UTR mut), was used to co-transfected MSCs together with as-miR-205-5p or null plasmids in a dual luciferase reporter assay. The luciferase activity was measured. HO: Hoechst 33342 staining for nuclei. *p < 0.05. NS: non-significant. *N* = 5.

### Preservation of MSC properties in as-miR-205-5p-transfected MSCs

Before we examined the effects of miR-205-5p-depletion in MSCs on their therapeutic potential in DF, we checked whether alteration of miR-205-5p levels may alter MSC property. We found that as-miR-205-5p-MSCs were able to be induced to differentiate into chondrocytes (Figure 4A), osteocytes (Figure 4B) and adipocytes (Figure 4C). Moreover, surface marker analysis for CD73, CD90, CD105, CD34, CD45 and HLA-DR in as-miR-205-5p-MSCs was consistent with an MSC phenotype (Figure 4D). Hence, transfection with as-miR-205-5p does not alter MSC properties.

**Figure 4:** Preservation of MSC property by as-miR-205-5p-transfected MSCs (**A**) Differentiation of as-miR-205-5p-MSCs into chondrocytes by Alcian blue staining. (**B**) Differentiation of as-miR-205-5p-MSCs into osteocytes by Von kossa staining. (**C**) Differentiation of as-miR-205-5p-MSCs into adipocytes by Oil red O staining. (**D**) Representative flow charts for CD73, CD90, CD105, CD34, CD45 and HLA-DR (red) in as-miR-205-5p-MSCs, compared to isotype controls (blue). Scale bars are 10 μm.

### Depletion of miR-205-5p in grafted MSCs does not reverse diabetes

Finally, we examined the effects of miR-205-5p-depletion in MSCs on their therapeutic potential in DF. NOD/SCID mice received STZ to induce diabetes. One week later, ulcers were generated in the right limb and the mice received intradermal transplantation of either mull-MSCs or as-miR-205-5p-MSCs at the ulcer site. The mice were followed up for 4 weeks before sacrifice and final analysis (Figure 5A). We found that STZ-treated mice developed sustained hyperglycemia within 1 week, and grafting with either null-MSCs or as-miR-205-5p-MSCs did not reserve hyperglycemia (Figure 5B), which were supported by beta cell mass quantification (Figure 5C), demonstrated by representative immunostaining images for insulin (Figure 5D).

**Figure 5:** Depletion of miR-205-5p in grafted MSCs does not reverse diabetes The effects of miR-205-5p-depletion in MSCs on their therapeutic potential in DF were examined. (**A**) Schematic of the model: NOD/SCID mice received STZ to develop diabetes. One week later, ulcers were generated in the right limp and the mice received intradermal transplantation of either mull-MSCs or as-miR-205-5p-MSCs at the site of ulcer. The mice were followed up for 4 weeks before sacrifice and final analysis. Group 1: untreated mice (UT: no STZ, no MSCs); group 2: STZ-treated mice (STZ; no MSCs); group 3: STZ+null-MSCs (STZ and transplanted with null-MSCs); group 4: STZ+as-miR-205-5p-MSCs (STZ and transplanted with as-miR-205-5p-MSCs). *N* = 10 in each group. (**B**) Fasting blood glucose (**C**) beta cell mass (**D**) Representative immunostaining images for insulin. Dashed circles indicated islets. NS: non-significant. *N* = 10. Scale bars are 100 μm.

### Depletion of miR-205-5p in grafted MSCs increases their therapeutic potential in DF

Next, we examined the effects of miR-205-5p depletion on wound healing from DF-associated ulcers. We found that the wound was completely cured in 4 weeks in untreated mice (UT; no STZ, no MSCs). The ulcer did not reduce in STZ-only treated mice. Transplantation of null-MSCs improved wound healing, but transplantation of as-miR-205-5p-MSCs on wound healing appeared to have more pronounced effects than transplantation of null-MSCs (Figure 6A). Vessel density was measured in mice 4 weeks after MSC transplantation. We found that the vessel density was significantly reduced by STZ treatment in the ulcer tissue. Transplantation of null-MSCs significantly increased vessel density, but the increases in vessel density by transplantation of as-miR-205-5p-MSCs appeared to be greater than transplantation of null-MSCs, shown by representative images (Figure 6B), and by quantification (Figure 6C). Thus, depletion of miR-205-5p in MSCs increases their therapeutic potential in DF.

**Figure 6:** Depletion of miR-205-5p in grafted MSCs increases their therapeutic potential in DF (**A**) Quantification of ulcer area in 4 groups, 4 weeks after MSC transplantation. (**B**–**C**) Quantification of vessel density in 4 groups, 4 weeks after MSC transplantation, shown by representative images (B), and by quantification (C). *p < 0.05. (red *: STZ+null-MSCs vs STZ; green *: STZ+as-miR-205-5p-MSCs vs STZ+null-MSCs). *N* = 10. Scale bars are 100 μm.

## DISCUSSION

Besides playing an essential role in embryonic development, MSCs are also actively involved in tissue regeneration in adulthood owing to their high competency and self-renewal properties [22]. Being an important stem cell population with adulthood accessibility renders MSCs a critical source for translational clinical applications [23]. Recent advances in gene editing create new approaches for regenerative medicine, and increase the prospect of application of MSCs. Indeed, Liu et al. showed that depletion of miR-937 significantly improved the therapeutic outcome in a mouse model for Alzheimer's disease mice, seemingly through augmentation of the levels of BDNF by loss of inhibitory effects of miR-937 [24]. Moreover, Yan et al. showed that expression of as-miR-548e recapitulated the effects of MSCs on collagen-induced mouse arthritis, likely through reactivation of IkappaB [25]. Furthermore, overexpression of miR-195 in human MSCs reduced osteogenic differentiation and enhanced cell proliferation through regulation of VEGF protein translation [26]. Very recently, VEGF has been found to be a target of miR-205-5p in glioma [20]. These reports encouraged us to start this study in searching for a way to improve the potential of MSC in treating DF through gene modification.

VEGF is a growth factor with complex mechanisms controlling its synthesis and release into extracellular matrix. Of note, previous studies have demonstrated that among all VEGF family members, VEGF-A (here simplified as VEGF) has the highest effects on re-vascularization associated with DF [10]. Moreover, among the three isoforms of VEGF, VEGF-165 is the most critical player [27, 28]. Hence in the scope of the current study, we focused on the study on it. We have recently shown that VEGF synthesis and release may be differentially regulated in pancreatic beta cells and duct cells [7]. Thus, the cellular storage of VEGF and release may be controlled by cell-specific mechanisms. Here, we analyzed both cellular VEGF and VEGF in the conditioned media to exclude the possibility that the differential levels of VEGF mRNA and protein in MSCs may result from the control of VEGF release in MSCs. We excluded this possibility and addressed an miRNA-regulated mechanism, since the half-life of VEGF is very short [8], and since there are reports of the presence of miRNA-mediated post-transcriptional control of VEGF [20, 26, 29, 30] but no evidence for its being regulated through protein modification like phosphorylation, acetylation and ubiquitination [31].

In the study that reported VEGF as a target of miR-205-5p in glioma [20], a different binding site on the 3′-UTR of VEGF mRNA from the current study was shown, suggesting the possible presence of different regulatory sites by miR-205-5p on the 3′-UTR of VEGF mRNA. It is thus interesting to experimentally compare the defined mutate sites in either experimental setting.

VEGF could be directly expressed in MSCs, rather than indirectly enhanced through a regulatory miRNA. However, we think that VEGF modification in the indirect way may be safer, more effective, and more translational. First, the body is very sensitive to changes in VEGF levels, since the physiological effects of VEGF are dosage-dependent over a very narrow physiologic range [31–34]. Direct overexpression of VEGF under a regular promoter may significantly increase its expression levels, leading to severe pathological situations, like bleeding. However, the changes in VEGF levels by miR-205-5p appeared to be modest, and physiologically sound. Second, direct expression of VEGF may further increase the levels of miR-205-5p in MSCs as a negative feedback, which substantially reduces the systemic efficiency, or even leads to occurrence of ER stress.

Here, we knocked down a highly expressed VEGF-antagonizing miRNA -miR-205-5p- in MSCs, which effectively increased VEGF and pro-angiogenic effects of MSCs. To the best of our knowledge, this is the first study to show that the therapeutic effects of MSCs on DF could be augmented through modification of a miRNA in MSCs. Compared to trophic factor infusion (e.g. here, injection of recombinant VEGF), a cell-based therapy (MSCs) has advantages like more sustained effects, better biological control, and fewer side effects. The results from the current study suggest that suppression of miR-205-5p in MSCs may be a promising strategy to increase their therapeutic potential in treating DF.

## MATERIALS AND METHODS

### Protocol approval

All the experimental methods in the current study have been approved by the research committee at the First Affiliated Hospital of Nanchang University. All the experiments have been carried out in accordance with the guidelines from the research committee at the First Affiliated Hospital of Nanchang University. All animal experiments were approved by the Institutional Animal Care and Use Committee at the First Affiliated Hospital of Nanchang University (Animal Welfare Assurance). Surgeries were performed in accordance with the Principles of Laboratory Care, supervised by a qualified veterinarian.

### Cell culture and differentiation of MSCs

Human endothelial cells (HUVEC) were purchased from American Type Culture Collection (ATCC, Rockville, MD, USA; Catalog number: CRL-1730), and were cultured in ATCC-formulated of F-12K Medium (ATCC; Catalog number: 30-2004) suppled with 0.1 mg/ml heparin, 0.03 mg/ml endothelial cell growth supplement and 10% fetal bovine serum (Sigma-Aldrich, St. Louis, MO, USA). Human bone-marrow derived MSCs were purchased from ATCC (Catalog number: PCS-500-012), and were cultured in bone marrow-derived MSC growth media (ATCC; Catalog number: PCS-500-041) suppled with MSC growth kit (ATCC; Catalog number: PCS-500-030) in a humidified chamber with 5% CO_2_ at 37°C. The MSCs were maintained in culture until reaching 80% confluence before splitting. The passage 5 was used for the current study.

Chondrogenetic differentiation assay of MSCs was performed using Chondrocyte Differentiation Tool (ATCC; Catalog number: PCS-500-051). Osteogenic differentiation assay of MSCs was performed using Osteocyte Differentiation Tool (ATCC; Catalog number: PCS-500-052). Adipogenic differentiation assay of MSCs was performed using Adipocyte Differentiation Toolkit for Adipose-Derived MSCs and Preadipocytes (ATCC; Catalog number: PCS-500-050). Two weeks after incubation in these differentiation media, Alcian blue staining, Von kossa staining and Oil red O staining were applied for differentiated chondrocytes, osteocytes and adipocytes, respectively.

### Genetic editing of human MSCs

The null or antisense for miR-205-5p (as-miR-205-5p) was cloned into a pCMV-DsRed-Express Vector (Catalog number: 632416; Clontech, Mountain View, CA, USA) backbone at the site between CMVp and red fluorescent protein (RFP). The human MSCs were transfected with 50 nmol/l plasmids using Lipofectamine 3000 (Invitrogen, St. Louis, MO, USA). The transfected cells expressed RFP, which allowed them to be purified by flow cytometry.

### Diabetic mice, DF and MSC transplantation

Diabetes was induced in 10-week-old male immune-deficient NOD/SCID mice (SLAC Laboratory Animal, Shanghai, China) by intraperitoneal injection of streptozotocin (STZ) at 130 mg/kg body weight, as has been described before [35]. One week later, the mice that had developed diabetes received induction of foot ulcer. Briefly, the dorsal portion of the right limb was shaved, cleaned and the area of the skin to be removed was marked before being cut off with a sterile fine scissor. A 0.5-mm-thick, 10-mm-inner-diameter silicone ring was placed around the wound. Wounds were monitored and wound dressings were changed every other day. The vertical and horizontal wound gaps were measured with vernier caliper. The wound gap was calculated as the average of vertical and horizontal wound gaps. Four weeks after development of diabetic ulcer, mice received intradermal injection of 10^6^ MSCs in 50 μl saline at the site of skin ulcer.

### Quantitative real-time PCR (RT-qPCR)

Total RNA were extracted using the miRNeasy mini kit (Qiagen, Hilden, Germany). Complementary DNA preparation and quantitative real-time PCR (RT-qPCR) were done, as have been described before [36]. All primers were purchased from Qiagen. Data were collected and analyzed using 2-ΔΔCt method. Values of genes were first normalized against GAPDH, and then compared to experimental controls.

### Western blot

Protein isolation and Western blotting were done, as has been described before [37]. Primary antibodies were rat anti-CD31 (Becton-Dickinson Biosciences, San Jose, CA, USA) and rabbit anti-GAPDH (Cell Signaling, Carpinteria, CA, USA). Secondary antibody is HRP-conjugated anti-rabbit or anti-Rat (Jackson ImmunoResearch Labs, West Grove, PA, USA). Blotting images were representative from 5 repeats. GAPDH was used as a protein loading control.

### Luciferase-reporter activity assay

The target gene of miR-365 was predicted by TargetScan, using the context++ score system, as has been instructed before [21]. The dual-luciferase reporter plasmids, p-3′-UTR-VEGF wt (containing the wild-type VEGF 3′-UTR binding site in luciferase reporter plasmid) and p-3′-UTR-VEGF mut (containing the mutant VEGF 3′-UTR) were constructed using p-3′-UTR-plasmid backbone (RiboBio Co. Ltd., Shanghai, China). For the luciferase assay, the p-3′-UTR-plasmid (wt or mut) was co-transfected with as-miR-205-5p plasmid into MSCs using Lipofectamine^TM^ 3000 Reagent (Invitrogen). Then the luciferase activity was analyzed using dual-luciferase reporter assay system (Promega, Shanghai, China), 48 hours after co-transfection.

### Flow cytometry

For characterization of MSC phenotype or purification of transfected MSCs, flow cytometry was performed as described before [38]. The antibodies are FITC-conjugated anti-CD73, CD90, CD105, CD34, CD45 and HLA-DR (Becton-Dickinson Biosciences). RFP and FTIC-lectin were detected by direct fluorescence.

### Fasting blood glucose, beta cell mass and vessel density

Fasting blood glucose has been described before [39]. Beta cell mass measurement has been described before [40]. For vessel density measurement, 50 μl FITC-lectin (Vectorlabs, Burlingame, CA USA) was injected via tail vein to the mice 5 minutes before sacrifice. The vessel density was determined as the ratio of lection+ area versus total area, as has been described before [7, 8].

### Histology and immunostaining

After FITC-lectin perfusion, mouse pancreas or limb skin tissue was dissected out and fixed in 4% paraformaldehyde (PFA, Sigma-Aldrich) for 6 hours. After overnight incubation in 30% sucrose, samples were frozen in liquid nitrogen and embedded in tissue freezing medium. Immunostaining has been done as described before [36].

### ELISA

The cellular and secreted levels of VEGF were determined in cell extracts or conditioned media, respectively, using VEGF enzyme-linked immunosorbent assay (ELISA; R&D System, Los Angeles, CA, USA), as has been described before [7, 8].

### Statistical analysis

All values represent the mean ± standard deviation (SD). Statistical analysis of group differences was carried out using a one-way analysis of variance (ANOVA) test followed by the Fisher's Exact Test to compare two groups (GraphPad Software, Inc. La Jolla, CA, USA). A value of *p* < 0.05 was considered statistically significant after Bonferroni correction.
